The article "Clinical Observation of Salvianolic Acid Combined with Panax Notoginseng Saponins Combined with Basic Nursing Intervention on Cerebral Ischemia-Reperfusion Injury in Rats" was published in 2022. Journal: J Healthc Eng.

# Clinical Observation of Salvianolic Acid Combined with Panax Notoginseng Saponins Combined with Basic Nursing Intervention on Cerebral Ischemia-Reperfusion Injury in Rats

**DOI:** 10.1155/2022/8706730

**Published:** 2022-01-30

**Authors:** Zhaopeng Zheng, Shanshan Liang, Shasha Sun, Pengfei Liu, Ling Yu

**Affiliations:** ^1^Health Management Department, Jiaozhou Central Hospital, Qingdao 266300, China; ^2^Department of Neurology (I), Affiliated Qingdao Central Hospital, Qingdao University, Qingdao 266042, China; ^3^Department of Neurosurgery, Affiliated Qingdao Central Hospital, Qingdao University, Qingdao 266042, China; ^4^Department of Neurology, Zhangqiu District People's Hospital, Jinan 250200, China; ^5^Department of Neurology, Yantaishan Hospital, Yantai 26400, China

## Abstract

**Objective:**

To analyze the clinical observation of salvianolic acid combined with panax notoginseng saponins combined with basic nursing intervention on cerebral ischemia-reperfusion injury in rats and its effects on the expression of apoptosis-related proteins Bcl-2, Bax and caspase-3.

**Methods:**

A total of 72 male Wistar rats were randomly divided into sham, ischemia/reperfusion (I/R), edaravone (Eda), salvianolic acid (SA), panax notoginseng saponins (PNS), and SA+PNS group. After administration for 5 days, the neurological function, cerebral infarction volume, brain index, and brain water content of rats were observed. ELISA kit assay was applied to measure the levels of IL-1*β*, IL-6, IL-8, TNF-*α*, MDA, SOD, GSH-Px, and T-AOC activity. Western blotting assay was used to detect the protein levels of p-53, NF-*κ*B, Bcl-2, Bax, and Caspase-3 in the brain tissues surrounding infarction lesion.

**Results:**

Compared with sham group, the mNSS score, brain index, brain water content, infarction volumes, MDA activity, and the levels of IL-6, IL-8, TNF-*α* and IL-1*β* as well as the protein levels of p-53, NF-*κ*B, Bax and Caspase-3 were significantly increased, while the levels of Bcl-2 protein, SOD, GSH-Px and T-AOC were significantly decreased in I/R group. However, these levels were reversed in SA group, PNS group and SA + PNS group. Moreover, these changes in SA + PNS group were more obvious than those in SA and PNS group, and the differences were statistically significant.

**Conclusions:**

SA, PNS and they combined with basic nursing have protective effects on cerebral I/R injury, and the combination with basic nursing has better effects than that used alone. The mechanism may be to regulate the expression of downstream apoptotic proteins by inhibiting the TLR4/NF-*κ*B signaling pathway, thereby reducing neurological damage in rats.

## 1. Introduction

Cerebral infarction, also known as cerebral ischemic stroke, is a common disease of the nervous system, which causes the obstruction or blockage of brain blood supply, resulting in oxygen and nutrient deficiency, irreversible damage to local brain tissue, leading to brain tissue ischemia and hypoxic necrosis [1]. Cerebral ischemia-reperfusion (I/R) injury refers to the restoration of blood supply after cerebral ischemia for a period of time. Although the ischemic organs and tissues can be regained with oxygen supply, the ischemic tissue damage and dysfunction are more severe, manifested by changes in hemodynamics, enlarged brain tissue infarct size, abnormal autophagy and apoptosis of nerve cells, etc. [2]. I/R is characterized by high morbidity, high disability rate, high mortality rate and low cure rate, which seriously affects the health and life of patients [3]. Clinically, timely restoration of brain blood supply and rescue of dying nerve cells is the key to the treatment of cerebral infarction. Recent studies [4] have confirmed that many clinical drugs have protective effects on cerebral I/R injury, mainly reflected in free radical scavenging, reducing intracellular calcium overload, inhibiting cell apoptosis, alleviating or preventing inflammatory reaction, etc. Clinical studies have found [5] that, compared with western drugs, Traditional Chinese medicine (TCM) has significant efficacy and fewer adverse reactions in the prevention and treatment of ischemic cerebrovascular diseases, with broad application prospects. TCM believes [6] that stroke and blood stasis are common pathological factors of cerebrovascular diseases. The main chemical components of salvia miltiorrhiza include water-soluble phenolic acids, such as salvianolic acid B, danshensu and rosinic acid, and lipid soluble diterpenoids, such as tanshinone and cryptotanshinone. The main active ingredient of panax notoginseng is the total saponins of panax notoginseng, which can improve the injury caused by cerebral ischemia and ischemia reperfusion, promote the recovery of nerve function, reduce the oxygen consumption of myocardium and improve the blood supply of myocardium [7, 8]. Clinically, salvia miltiorrhiza and panax notoginseng are commonly used as a pair of blood-activating drugs, which complement each other and are widely used in the treatment of cardiovascular and cerebrovascular diseases [9]. Studies have found [10] that the combination of salvianolic acid and panax notoginseng saponins can reduce cerebral I/R injury by reducing the volume of cerebellar infarction, alleviating oxidative stress injury and reducing inflammatory response. Studies have found [11] that apoptosis is one of the important mechanisms of cerebral I/R injury. Apoptosis is involved in the pathological process of many diseases and is closely related to the pathological mechanism of cerebral I/R injury. Among them, the pro-apoptotic protein Bax and the anti-apoptotic protein Bcl-2 are dynamic *in vivo* and participate in the regulation of apoptosis together [12]. As an important member of the Caspase family, Caspase-3 mediates the protease cascade of apoptosis and is the common downstream effect part of various apoptosis pathways [13]. In this study, we investigated the neuroprotective effects of salvianolic acid combined with panax notoginseng saponins on cerebral I/R injury in rats and the effects of apoptosis related proteins Bcl-2, Bax and caspase-3.

## 2. Materials and Methods

### 2.1. Drugs and Reagents

SA were purchased from Tianjin Tasly Zhijiao Pharmaceutical Co., Ltd. (approval number: National Medicine Zhunzi Z20110011); PNS was purchased from Yunnan Teana Pharmaceutical Co., Ltd. (approval number: Z53020178); Eda was purchased from Sinopharm Group Guorui Pharmaceutical Co., Ltd. (specification 20 mL/30 mg, approval number: National Medicine Standard H20080056); SOD, MDA, GSH-Px and T-AOC detection kits were purchased from Shanghai Hengyuan Biotechnology Co., Ltd.; Chloral hydrate was purchased from Wuhan Huaxiang Kejie Biotechnology Co., Ltd.; None Hydroethanol was purchased from Chengdu Chemical Reagent Factory; Nitrogen chloride phenyltetrazolium (TTC) was purchased from Hubei Bojie Biotechnology Co., Ltd.; TNF-*α*, IL-6, IL-8, IL-1*β* kits were purchased from Wuhan Huamei Bioengineering Co., Ltd.; Bcl-2, Bax, Caspase-3, NF-*κ*B p53 and NF-*κ*B p53 primary antibodies. The secondary antibodies such as horseradish peroxidase (HRP) goat anti-rabbit IgG and HRP goat anti-mouse IgG were purchased from American Thermo Company.

### 2.2. Experimental Animals

72 SPF-grade healthy male Wistar rats, weighing (270 ± 20) g, were provided by Beijing Weitong Lihua Laboratory Animal Technology Co., Ltd. (animal license number: SCXK (Beijing) 2020-0016). They were raised in separate cages, with a breeding temperature of 20-25 °C and a relative humidity of 50%-65%. The animal experiment was approved by the Animal Care and Use Committee of Yantaishan Hospital (approval no. 201906035). The experimental rats were allowed to eat and drink freely, and the utensils and litter were changed every day.

### 2.3. Main Instrument

The microplate reader was purchased from Shandong Brocade Bio-Industry Co., Ltd., the refrigerator was purchased from Jinan Alabao Instrument Equipment Co., Ltd., the constant temperature water bath was purchased from Zhejiang Haining Medical Equipment Factory, the high-speed refrigerated centrifuge was purchased from Germany Sigma, the fluorescence quantitative PCR instrument was purchased from Jinan Alchemy Instrument Co., Ltd., the electronic balance was purchased from Zhengzhou Pushton Electronic Equipment Co., Ltd., the cryogenic centrifuge (3-5w type) was purchased from Jiangsu Huada Centrifuge Manufacturing Co., Ltd., the upright metallographic microscope (SG-51 type) was purchased from Shanghai Optical Instrument Factory, Protein electrophoresis and transfer membrane instrument was purchased from Bio-Rad, USA.

### 2.4. Grouping and Administration

72 Wistar rats were divided into 6 groups by the random number method, namely sham group, I/R group, Eda group, SA group, PNS group, and SA+PNS group, with 12 cases in each group. They were administered by tail vein injection, of which Eda group, SA group and PNS group were given 6 mg/kg, 21 mg/kg and 100 mg/kg once a day for 5 consecutive days, respectively. The sham group and I/R group were given the same volume of normal saline. All rats were given consistent basic care. The intraoperative body temperature of rats was generally maintained at (37 ± 0.5) °C and the room temperature was kept at 24 °C ∼ 26 °C.

### 2.5. Preparation of Rat Cerebral Ischemia/Reperfusion Injury Model

The middle cerebral artery occlusion/reperfusion model (MCAO/R) was established by the suture method. After the rats were anesthetized by inhalation of isoflurane, the cerebral blood flow was monitored by a laser doppler flowmeter, the common carotid artery (CCA), external carotid artery (ECA) and internal carotid artery (ICA) were bluntly separated from the center of the neck. The thread plug was insert from the ECA to the ICA through the CCA bifurcation to block the blood supply of the middle cerebral artery. After embolization for 1.5 hours, the thread plug was pulled out and reperfusion was completed. In the sham operation group, only the neck vessels were exposed, and the suture plug was not treated.

### 2.6. Observation Indicators and Evaluation Methods

(1) Neurological deficit score: After 5 days of reperfusion, the rats are evaluated for neurological deficit according to Zea-longa 5 score [14]. The specific scoring rules include spontaneous activity, forelimb movement, climbing ability, somatosensory, beard stimulation, balance beam experiment, and statistics. (2) Determination of cerebral infarction volume: After the neurological function score, the rats in each group were decapitated under anesthesia to remove the olfactory bulb, cerebellum, and brainstem and then placed in a refrigerator at -20 °C for 30 min. The brain were cut into 2 mm thick coronal sections, and put in 2% TTC phosphate buffer solution for 30 min at 37 °C and in 10% formaldehyde solution for 2 h in the dark. The normal brain tissue was red, and the cerebral infarction was white. A computer image analysis program was used to scan all the brain slice images to determine the area of the cerebral infarction area. The ratio of infarct volume [15] (the sum of the infarct area of all brain slices × the thickness of the brain slice) and cerebral infarction volume (infarct volume/whole brain volume×100%) was calculated. (3) Determination of brain index and brain water content: After 5 days of reperfusion, the rats were anesthetized and decapitated, and the brains were taken out and weighed. Brain index = wet brain weight (g)/body weight (100 g), brain water content (%) = [wet brain weight (g)-brain stem weight (g)]/wet brain weight (g)×100% [16] . (4) Determination of stress indicators: 10% of the brain tissue was crushed and homogenized with lysate precooled at 4 °C, and then centrifuged at 3 000 r/min for 15 min. The supernatant was taken and the MDA content and t-AOC, SOD and GSH-Px activities were determined according to the kit operating instructions. (5) Determination of inflammatory factors in brain tissue: 10% of the brain tissue was crushed and homogenized with lysate precooled at 4 °C, and then centrifuged at 3 000 r/min for 15 min. The supernatant was taken and the tumor Necrosis factor-*α* (TNF-*α*), interleukin-1*β* (IL-1*β*), interleukin-6 (IL-6) and interleukin-8 (IL-8) were detected by the kit instructions. (5) Western blotting method to detect protein expression levels: The brain tissues were taken out and then digested with trypsin. The total protein was extracted and then performed electrophoresis. After transferred onto membranes, the proteins were blocked and incubated with primary antibodies (Bcl-2, Bax, Caspase-3, NF-*κ*B) overnight, followed by the secondary antibody for 2 h. The absorbance analysis was performed to calculate the expression of each protein relative to the internal reference protein *β*-actin.

### 2.7. Statistical Analysis

The SPSS 20.0 statistical software (IBM, NY, USA) was used for statistical analysis of the data. The measurement data was expressed as (x ± s) of three independent experiments, and the data comparison between groups was performed by t test. The difference is statistically significant with p < 0.05.

## 3. Results

### 3.1. The Effect on the Neurological Deficit Score of Rats

Compared with the sham group, the mNSS score of the I/R group was significantly higher, the neurological deficit was serious, and the difference was statistically significant (^∗^p < 0.01). Compared with the I/R group, the mNSS score of SA group, PNS group and SA + PNS group was significantly decreased (^∗∗^p < 0.01), and the mNSS score of SA + PNS group was significantly lower than that of SA group and PNS group, the difference was statistically significant (^#^p < 0.01). There was no statistically significant difference in mNSS scores between the Eda group and the SA+PNS group (p>0.05) are shown in Figure 1.

### 3.2. The Effects on Cerebral Infarction Volume and the Expressions of p-53 and NF-κB in the Brain Tissue around the Infarct Focus in Rats

Compared with the sham group, the cerebral infarction volume and the protein levels of p-53 and NF-*κ*B in the brain tissues around the infarct were significantly increased in the I/R group, and the difference was statistically significant (^∗^p < 0.01). Compared with the I/R group, these above were significantly decreased in the SA group, PNS group, and SA + PNS group (^∗∗^p < 0.01), and the volume of cerebral infarction and p-53 and NF-*κ*B levels in SA+PNS group was significantly lower than that of SA group and PNS group, the difference was statistically significant (^#^p < 0.01). There was no statistically significant difference in the SA+PNS group and Eda group (p>0.05), as shown in Figure 2 and Table 1.

### 3.3. The Effects on the Brain Index and Brain Water Content of Rats

Compared with the sham group, the brain index and brain water content of rats in the I/R group was increased significantly (^∗^p < 0.05). Moreover, compared with the I/R group, the brain index and brain water content of rats in the SA group, PNS group and SA + PNS group were decreased significantly (^∗∗^p < 0.05), and the brain index and brain water content of rats in the SA+PNS group were significantly lower than those in the SA group and the PNS group. The difference was statistically significant (^△^p < 0.05), as shown in Table 2.

### 3.4. The Effects on the Activities of MDA, SOD, GSH-Px, and T-AOC in Rat Brain Tissue

Compared with the sham group, the content of MDA in the brain tissue of rats in the I/R group was significantly increased, and the content of SOD, GSH-Px and T-AOC was significantly decreased, and the difference was statistically significant (^∗^p < 0.01). Compared with I/R group, MDA content were decreased significantly, while the SOD, GSH-Px and T-AOC content were increased significantly in SA, PNS and SA+PNS groups (^∗∗^p < 0.05), Moreover, the MDA, SOD, GSH-Px and T-AOC content in SA+PNS group were more obvious than that of SA and PNS groups, and the difference was statistically significant (^#^p < 0.05), as shown in Figure 3.

### 3.5. The Effects on the Expression of IL-6, IL-8, TNF-*α*, and IL-1*β* in Rat Brain Tissue

Compared with the sham group, the expressions of IL-6, IL-8, TNF-*α* and IL-1*β* in the brain tissue of the I/R group were increased significantly (^∗^p < 0.01). Compared with the I/R group, the expressions of IL-6, IL-8, TNF-*α*, and IL-1*β* in the brain tissue of rats in the SA, PNS and SA+PNS groups were significantly decreased (^∗∗^p < 0.01), and these levels in the SA+PNS group were decreased more significantly than those in the SA and PNS groups (^#^p < 0.01), as shown in Figure 4.

### 3.6. The Effects on the Levels of Bcl-2, Bax, and Caspase-3 in Rats

Compared with the sham group, the level of Bcl-2 in I/R group was significantly decreased, while Bax and Caspase-3 levels were increased significantly (^∗^p < 0.01). Compared with the I/R group, the level of Bcl-2 was increased significantly, while Bax and Caspase-3 levels were decreased significantly in the brain tissue of SA, PNS and SA+PNS group (^∗∗^p < 0.05). Moreover, these levels in SA+PNS group changes more significantly than those in SA and PNS groups (^#^p < 0.01), as shown in Figure 5.

## 4. Discussion

Cerebral I/R injury is a neurological disease that provides timely blood supply support when the blood supply of tissues and organs is insufficient. Eventually, a series of complex structural damage and dysfunction appear due to the interaction of multiple mechanisms and multiple links. Apoptotic necrosis is one of the important links of cerebral ischemia reperfusion injury [17]. It is a serious threat to human health. Most patients with ischemic cerebrovascular disease need care because of sequelae such as intellectual and limb dysfunction. The increasing number of such patients has become a very important medical and social problem. Studies believe that [18] timely restoration of blood supply to the cerebral ischemic area and reduction of nerve cell damage are the key to the treatment of cerebral I/R injury. TCM has the advantages of multi-component, multi-target, small side effects, stable curative effect, etc., and it has attracted more and more attention in the treatment of cerebral ischemia. Ischemic cerebrovascular disease belongs to the category of “stroke disease“ in Chinese medicine. It is clinically manifested as confusion, dizziness, hemiplegia, crooked mouth and eyes, slurred speech and other symptoms. This disease is characterized by liver and kidney yin deficiency, Qi and blood deficiency and blood stasis are blocked, so the treatment should be based on nourishing yin and promoting blood circulation, resolving phlegm and dredging collaterals [19]. SA was first seen in “Shen Nong's Materia Medica“, which has the effect of promoting blood circulation and removing blood stasis, and PNS has the power of promoting blood circulation and removing blood stasis, tonic and strong [20, 21]. During the experiment, the vital signs of rats were closely monitored, and abnormal changes were dealt with in time. In the perioperative period, heat preservation measures were taken to prevent the body from harming the body due to low body temperature. Postoperative care is also very important. Effective anti-inflammatory care for surgical wounds is of positive significance for preventing postoperative infections.

After the reperfusion of cerebral ischemia patients restores the blood supply, brain tissue cells are damaged and the cells rupture, the water overflow in the cells causes the brain water content to increase, and the nerve function is affected [22]. This study showed that compared with the I/R group, the neurological damage score, brain index and brain water content in the SA, PNS and SA+PNS groups were decreased, and the SA+PNS group decreased more significantly (p < 0.05), indicating that the combination of SA and PNS combined with basic nursing care can effectively alleviate the brain I/R injury, and can effectively reduce the neurological damage, cerebral infarction volume, p-53 level, brain index and brain water content around the infarct area after ischemia perfusion in rats, which means that the combination of the two prescriptions has a good protective effect on cerebral ischemia. MDA is one of the end products of the lipid peroxidation reaction caused by oxygen free radicals, which can cause degeneration and damage of cell membranes and reduce the fluidity and permeability of cell membranes. The content of MDA indirectly reflects the degree of tissue damage by free radicals [23]. Both SOD and GSH-Px are antioxidant enzymes in the body. SOD can effectively remove superoxide anion free radicals in the body, reduce free radical damage, repair the blood-brain barrier, increase permeability, and reduce cerebral edema [24]. GSH-Px can block lipid peroxidation to reduce cell damage caused by oxygen free radicals, reduce MDA levels, and reduce brain tissue cell membrane damage [25]. The detection of T-AOC can reflect the body's ability to resist peroxidation injury after acute cerebral ischemia and reperfusion, and can also be used to assess the degree of brain tissue peroxidation injury [26]. Modern pharmacological studies have shown that [27] PNS can promote the repair of glial cells, neurons and capillaries after cerebral I/R by increasing the activity of SOD and GSH-Px in the body and reducing the level of MDA. This study found that compared with I/R group, the levels of SOD, GPX, and T-AOC in rats treated with SA+PNS increased, and the content of MDA decreased significantly. It shows that SA+PNS can effectively inhibit oxidative stress. This may be because SA and PNS contain polyphenol compounds. These polyphenol compounds have strong antioxidant properties and effectively alleviate the stress in the brain tissue of I/R rats. The oxidation reaction alleviated I/R damage in rats. NF-*κ*B is widely present in eukaryotic cells and can regulate the release of a variety of immune inflammatory mediators, change the microenvironment of tumor growth, and regulate tumor cell proliferation, apoptosis and other processes [28]. Studies have shown [29] that the activation of the NF-*κ*B signaling pathway can also regulate the expression of apoptosis-related proteins Bcl-2, Bax, and Caspase-3, and induce cell apoptosis. This study found that compared with the I/R group, the expression of NF-*κ*B, Bax, and Caspase-3 in the brain tissue of the SA+PNS group were decreased and the Bcl-2 protein expression was increased. It shows that SA+PNS can inhibit the expression of NF-*κ*B, inhibit the TLR4/NF-*κ*B signaling pathway and affect the expression of downstream apoptosis-related genes, protect rat brain nerve cells from apoptosis after ischemia, and alleviate I/R damage . Studies have shown that [30, 31], SA acid and PNS can inhibit the TLR4/NF-*κ*B signaling pathway, and this study are basically consistent with them. There is an evidence that [32] inflammatory response mediates secondary brain injury after cerebral I/R. The inflammatory response after ischemia is mediated by many inflammatory factors, such as TNF-*α*, IL-6, IL-8 and IL-1*β*, among which TNF-*α*is especially important in cerebral I/R injury [33–35]. The results show that SA+PNS can effectively reduce the expression of TNF-*α*, IL-6, IL-8 and IL-1*β* inflammatory factors after cerebral I/R injury, and reduce the inflammatory response to brain tissue after reperfusion.

In summary, the combination of SA combined with PNS combined with basic nursing has a significant protective effect on the brain tissue of rats with cerebral I/R injury. It can significantly reduce the cerebral infarction volume of rats with cerebral I/R injury, improve brain edema, enhance the antioxidant activity of SOD, GSH-Px, and T-AOC, reduce MDA lipid peroxidation damage and inhibit the apoptosis of I/R rat brain cells and alleviate brain I/R injury through suppressing TLR4/NF-*κ*B signaling.

## Figures and Tables

**Figure 1:** Comparison of neurological deficit scores of rats in each group. ^∗^p<0. 01 vs sham; ^∗∗^p < 0.01 vs I/R; ^#^p < 0.01 vs SA or PNS.

**Figure 2:** Comparison of infarct volume of rat brain tissue in each group. ^∗^p < 0.05 vs sham; ^∗∗^p<0.01 vs I/R; ^#^p < 0.01 vs SA or PNS.

**Figure 3:** The effects of SA+PNS on the activities of MDA, SOD, GSH-Px and T-AOC in brain tissue (a) Comparison of MDA content in the brain tissue of each group of rats. (b) Comparison of the SOD content in the brain tissue of each group of rats. (c) Comparison of the GSH-Px content in the brain tissue of each group of rats. (d) Comparison of T-AOC content in the brain tissue of each group of rats. ^∗^p < 0.05 vs Sham; ^∗∗^p < 0.01 vs I/R; ^#^p < 0.01 vs SA or PNS.

**Figure 4:** The effect of SA+PNS on the expression of IL-6, IL-8, TNF-*α* and IL-1*β* in the brain tissue of each group of rats. (a) Comparison of the expression level of IL-6 in the brain tissue of each group. (b) Comparison of the expression level of IL-8 in the brain tissue of each group. (c) Comparison of the expression level of TNF-*α* in the brain tissue of each group. (d) Comparison of IL-1*β* expression levels in the brain tissue of rats in each group. ^∗^p < 0. 05 vs sham; ^∗∗^p < 0. 01 vs I/R; ^#^p < 0. 01 vs SA or PNS. The effects on the levles of Bcl-2, Bax and Caspase-3 in rats.

**Figure 5:** The effect of Danshen combined with Panax notoginseng on the expression of Bcl-2 protein, Bax protein and Caspase-3 protein in each group of rats. (a) Comparison of Bcl-2 protein expression levels of rats in each group. (b) Comparison of Bax protein expression levels of rats in each group. (c) Comparison of Caspase-3 protein expression levels of rats in each group. ^∗^p < 0.05 vs sham; ^∗∗^p < 0.01 vs I/R; ^#^p < 0.01 vs SA or PNS.

**Table 1:** Comparison of p-53 and NF-*κ*B protein expression in brain tissue around infarcted focus of rats in each group.

Group	*n*	p-53	NF-*κ*B
Sham	12	0.53±0.24	0.36±0.12
Eda	12	0.98±0.28	0.93±0.24
I/R	12	1.56±0.47	1.45±0.23
SA	12	1.31±0.36	1.24±0.28
PNS	12	1.28±0.33	1.26±0.31
SA+PNS	12	0.92±0.22	0.88±0.17
*t*_0_		12.334	14.652
*t*_1_		7.421	6.710
*t*_2_		10.106	8.634
*t*_3_		0.783	0.537
*P*_0_		<0.01	<0.01
*P*_1_		<0.05	<0.05
*P*_2_		<0.01	<0.01
*P*_3_		>0.05	>0.05

*t*_0_, *P*_0_, sham vs I/R; *t*_1_, *P*_1_, I/R vs SA; *t*_2_, *P*_2,_ SA vs SA+PNS; *t*_3_, *P*_3_, Eda vs SA+PNS.

**Table 2:** Effects of SA combined with PNS on brain index and water content of rats in each group.

Group	n	Brain index (g/100 g)	Wet weight (g)	Dry weight (g)	Water content (%)
Sham	12	0.48 ± 0.023	0.652 ± 0.021	0.147 ± 0.004	69.21 ± 2.23
Eda	12	0.52 ± 0.025^∗∗^	0.683 ± 0.028	0.148 ± 0.006	73.65 ± 3.12^∗∗^
I/R	12	0.63 ± 0.036^∗^	0.722 ± 0.036	0.150 ± 0.007	82.04 ± 3.24∗
SA	12	0.58 ± 0.032^∗∗^	0.706 ± 0.032	0.149 ± 0.005	77.81 ± 2.47^∗∗^
PNS	12	0.59 ± 0.031^∗∗^	0.702 ± 0.033	0.149 ± 0.006	78.23 ± 2.66^∗∗^
SA+PNS	12	0.54 ± 0.026^∗∗^^△^	0.675 ± 0.031	0.148 ± 0.004	72.14 ± 2.82^∗∗^^△^

^∗^P < 0.05 vs sham, ^∗∗^P < 0.01 vs I/R, ^△^*P < 0.05 vs SA or PNS*

## Data Availability

Data to support the findings of this study are available on reasonable request from the corresponding author.
